# Application of Neural Network Model Based on Multispecies Evolutionary Genetic Algorithm to Planning and Design of Diverse Plant Landscape

This article has been retracted.

**DOI:** 10.1155/2021/9031366

**Published:** 2021-10-18

**Authors:** Yuqiang Wu, Weiwei Guo, Dinghai Yang

**Affiliations:** ^1^Hainan College of Economics and Business, Haikou 571127, China; ^2^College of Forestry, Hainan University, Haikou 570228, China

## Abstract

In order to explore the feasibility of applying neural network model to landscape planning, based on the multispecies evolutionary genetic algorithm, a neural network model is proposed in this paper for the system design of diverse plant landscape planning. From the perspective of plant species diversity, this paper discusses landscape planning based on a neural network model. This landscape plan involves more than 180 plant species, mainly shrubs, fungi, and so on. The application of multispecies evolutionary genetic algorithm to landscape planning and design and the application of gene level coding and multispecies parallel evolution strategy to the evolutionary design of neural network have guiding significance for plant landscape planning and design. Compared with the traditional neural network modeling method and genetic algorithm, the proposed method has the advantages of wide network structure search space and simple algorithm calculation and design, independent of specific application background, and has strong application and promotion value. This method makes the model performance evaluation index more comprehensive and accurate and the model solution more reasonable. At the same time, combined with the specific status and corresponding changes of various plants in each season, this paper designs a targeted plan to rationally plan the specific spatial layout of the plant landscape and the combination of different types of plant landscapes, so as to effectively improve the quality of the landscape.

## 1. Introduction

The concept of urban development in China has been constantly updated, and the urbanization road with ecological civilization construction as the development route has been supported and achieved good results in practical development. The construction of modern landscape architecture is to achieve unified and harmonious ornamental and entertainment purposes by integrating related buildings, plants, regional landforms, water bodies, and other cultural and natural landscapes, provide a more comfortable and relaxing place for people's life and entertainment, and regulate the overall ecological situation of the city [1–3]. In the actual process of landscape architecture construction, designers tend to design a large number of plant landscapes, which can effectively enrich the beauty and harmony of the garden, and plant landscape design can also improve the overall aesthetic level of the garden. In such a design environment, it is necessary to strengthen the in-depth study of plant landscape planning and design, to provide a scientific basis for its integration into landscape architecture, and to bring new design features for urban construction. At present, the landscape architecture in different cities in China has its own characteristics, and the important factor of this differentiation is the different plant landscape design. The garden landscape planning and design of a variety of plant landscapes can be pleasing to the eye and provide people with good leisure activities; this is an important benefit of plant landscape planning and design. Under the background of China's deepening economic development, urban environmental construction is also more and more valued by people. Good landscape architecture can add luster to urban construction and improve people's living happiness [4, 5]. Under the double pressure of social pressure and the pace of life, people are in great need of places for entertainment and relaxation. The construction of landscape architecture is also to meet this need and bring people a sense of leisure and relaxation through plant landscape. At the same time, plant landscape planning and design are widely used in landscape architecture [6], which can effectively reduce urban air pollution and contribute to urban environmental ecological construction.

In order to reflect the overall unity and coordination of various landscape construction of landscape architecture, the relevant planning and design should fully combine the customs and geomorphology of the region, adopt the design method in accordance with local conditions, and carry out detailed planning and design on the basis of the local climate and geomorphology. To integrate plant landscape planning and design into landscape architecture, it is necessary to reflect the harmony between the two under the principle of overall unity, so as to provide a reference for the authenticity and feasibility of relevant design and planning [7–9]. When planning and designing the plant landscape of landscape architecture, we should use the strategy of conceptual planning, analyze the status quo of prebuilt landscape architecture through conceptual planning, set the planning and design goals of landscape architecture, combine these goals to do a good job in the multidimensional planning and design of landscape architecture, and design more details of landscape architecture accordingly. Landscape architects should be clear about the requirements and regulations of planning and objectives and do a detailed and multidimensional conceptual design of plant landscape according to the planning. Overall, it covers feature planning, time planning, and space planning. First, regarding feature planning, in the process of conceptual planning of plant landscape, characteristic planning is a key content. Designers should design featured landscapes in combination with the overall planning of landscape architecture and highlight the overall characteristics of various plant landscapes and landscape architecture on the whole, so as to present a more ideal design effect [10]. Second, regarding time planning, optimized time planning is of great significance in the design of plant landscapes. Combining the specific status and corresponding changes of various plants in each season, a targeted plan is designed, which can adapt to different seasons and present plant landscapes of different colors, thereby enhancing the practicality and ornamentalness of plant landscapes. Thirdly, regarding space planning, from the perspective of space planning, plant landscape construction space usually occupies a large area in landscaped gardens [11]. Therefore, it is necessary to reasonably plan the specific space layout of plant landscape and the collocation of different types of plant landscape to effectively improve the design quality of landscape architecture.

In the planning and design of landscapes, designers often choose to present specific design schemes by applying more intuitive design drawings. In the past for a long time, because of the limitations of technology, in the garden design, the design can only be hand painted and other ways to express the relevant design scheme require more time, and it is difficult to modify the scheme. The garden design assisted by a genetic algorithm greatly improves the efficiency and quality of design and effectively reduces the cost. The genetic algorithm is generally used for connection weight optimization and structure optimization of the neural network [12]. The structure optimization of the neural network is obviously a “multipeak” problem, the simple genetic algorithm is not effective in solving this problem, and the parallel genetic algorithm is one of the better improved methods. According to the modern genetics theory, the genetic information of organisms is contained in the genetic gene of the organism. In addition to the genetic information representing the characteristics of an individual, it also includes the genetic information of the characteristics of the species to which the individual belongs. Biological genes are divided into two parts: one part is called individual genes, reflecting the individual characteristics of the organism, and the other part, called the species gene, corresponds to the species attribute of the organism and controls the structure and some attributes of the individual gene. The difference of biological species is expressed as the difference of species gene from gene. Individuals of the same species have the same species genes, and their individual differences are reflected in the differences of individual genes [13]. Evolution at the individual level of organisms is represented by the optimization of individual genes within the same species, while evolution at the species level is represented by the optimization of species genes between different species. Based on the above theory, a multispecies evolutionary genetic algorithm is proposed, which can be applied to the structure learning of neural networks. The application of multispecies evolutionary genetic algorithm to landscape planning and design and the application of gene level coding and multispecies parallel evolution strategy to the evolutionary design of neural network have guiding significance for plant landscape planning and design.

## 2. Related Work

Since the concept of diverse plant landscape planning was proposed, scholars from different countries have conducted extensive discussions. Research on the compilation of urban flora and fauna diversity, spatial distribution, and habitat mapping began in the 1960s in Western Europe (Germany, Britain, and the Netherlands), North America (the United States), and Japan (The United States). Chen [14] believes that sustainable urban development should make rational use of its own resources, improve utilization efficiency, and focus on long-term development. In recent years, foreign studies have paid more attention to urban social environmental factors, such as the impact of population density, cultural characteristics of residents, and economic income on animal and plant diversity [15, 16]. The impacts of plant distribution and diversity on landscape planning were studied from landscape and local levels [17, 18]. At the same time, attention has also been paid to the impact of urban animal and plant diversity on human physical and mental health [7, 19]. Related scholars discussed how to build an animal and plant diversity protection system in the urban environment [19–22]. Part of the research has been focusing on the relationship between human daily activity interference and plant planting distance [23]. The study of plant diversity can be carried out in all kinds of urban land use.

With further development of social economy and urban construction, people's understanding of urban landscape construction is further deepened. A good urban environment is the unity of the overall environment and the change of local buildings and establishes a hierarchical structure integrating plants, landscapes, and human activity areas. In addition, many scholars began to study the theory of plant landscape ecology. Various researchers have conducted species cataloging and diversity comparative studies [23, 24] on plant diversity in urban built-up areas and natural mountains within the city. The types of urban green space include park green space, green isolation zone, residential green space, ancillary green space, and street green space. Research shows that, in the actual landscape design and construction process, in the initial stage of plant landscape planning and design, it is necessary to fully demonstrate the scientific rationality of plant landscape planning and design, in order to ensure that in the subsequent actual construction with operability. In the design act, the actual needs for relevant landscape architecture projects should be combined with specific design concepts, in order to obtain the best appreciation effect of plant landscape. At the same time, in the production of the program, we should pay enough attention to the reasonable layout of related landscape plants, the selection of plant types, the performance space of plants, and the coordination research with the surrounding areas, so as to improve the comprehensiveness and operability of the program design. In a word, plant landscape design is to fully combine the various design elements of landscape architecture and comprehensive consideration, so as to get the optimal planning and design scheme.

This paper attempts to discuss the problem of landscape planning based on a neural network model from the perspective of plant species diversity. A good plant landscape is conducive to beautifying the ecological environment of a landscaped garden, displaying the garden style, improving the living atmosphere, and providing leisure and entertainment. It is necessary to adhere to the correct concept of plant landscape design, optimize the design strategy, and design diversified plant landscapes that are compatible with the local customs, geographical environment, climate, and geology. It is also necessary to fully integrate the excellent cultural elements of traditional construction and design of landscape architecture. Through the proper collocation and reasonable selection of different plants, the cultural taste, practical effect, and aesthetic degree of landscape architecture can be effectively strengthened. This paper analyzes the diversity of plant landscape planning and hopes to be helpful to related workers.

## 3. Diverse Plant Landscape Planning Based on Neural Network Model

### 3.1. Landscape Area Selection and Planning Methods

The landscape planning area is selected to be located at a site on the outskirts of Beijing. Located at the northern end of the North China Plain, surrounded by the Taihang and Yanshan mountains from the north, northwest, and west, Beijing enjoys a humid continental climate and is influenced by monsoons. The East Asian monsoon makes summers wet, but winters are cold, dry, and windy due to the cold air from Siberia. Spring and autumn last for a short time in the four seasons. The average annual rainfall is 494.5 mm, mainly in summer. The average temperature is −2.9°C in January and 27.1°C in July. The natural vegetation is coniferous and broad-leaved mixed forest.

In this landscape design, architecture is the hardware, greening is the software, waterscape is the network, sketch is the node, and various professional technical means are adopted to assist the implementation of the design scheme. It covers areas such as regional, new town, neighborhood and community planning, park and recreation planning, transportation planning, campus planning and design, landscape renovation and restoration, heritage conservation, garden design, recuperation, and other special purpose areas. The composition should always revolve around fulfilling all the functions of the idea. In this, the main attention should be paid to the relationship between man and nature. In order to gradually enter the ideal realm of different sceneries, various methods are used in landscape construction to express nature, so as to achieve natural, indifferent, quiet, and implicit artistic effects. Modern landscape design ideas also advocate the harmony between people and nature. The goal and work of a landscape architect is to make people, buildings, communities, urban life, and the earth's ecology live in harmony. Landscape design composition includes two aspects: plane composition combination and three-dimensional modeling combination. The plane composition is mainly to express the traffic road, green area, and facility location in the form of plane diagrams in proportion and accurately. See Figure 1 for the composition of the elements in this plane composition.

### 3.2. Neural Algorithm Model Based on Multispecies Evolutionary Genetic Algorithm

As a learning tool of neural network, genetic algorithm is one of the most important research directions at present. As mentioned above, a simple genetic algorithm can solve the weight learning problem well, but it is not ideal for structure learning, which is not convenient for structure learning and weight learning at the same time. In this paper, neural network model based on multispecies evolutionary genetic algorithm is applied to multispecies plant landscape planning and design.

The different external characteristics of different populations are determined by the different genes of their populations. Population as a whole, through interpopulation hybridization, fusion, mutation, and new population, may also be due to survival of the fittest and die out. The hybridization and variation of individual organisms generally occur only within the same population. In addition to the fitness of a species, it also has its evolutionary ability to measure the merits of a species. The strategy of “species replacement” is to eliminate the species that do not meet the requirements and have poor evolutionary ability and replace them with new species. For newly created species, in order to prevent them from being eliminated before full evolution, “juvenile conservation” mechanism is set up. The total population size of all species remains constant during the evolution of the species layer. However, the population size is determined by the evolution of the most recent species during the evolution of individual layer, and the population size is not changed by the operation of individual layer evolution. The exchange operation follows the principle of “intraspecious exchange,” that is, the crossover occurs between individuals of the same species.

Neural network performance evaluation includes many factors such as network training error, network learning ability, network structure complexity, and network generalization ability. For example, for THE MLP with *P* learning sample groups, the training error [5] is

(1) $$\begin{array}{c} E=\frac{1}{P}\sum_{m=1}^{P}\sum_{i=1}^{N}{\left(Y_{i}^{N}-Y_{j}\right)}^{2}. \end{array}$$

For MLP, this generally means optimizing node weights without changing its network structure. In MLP structure learning, the individual evolution ability of species generally takes its optimal individual learning efficiency. In generation *T*, if *F*^*T*^ is the species fitness at the time of cycle *T*, MLP learning efficiency function [12] is

(2) $$\begin{array}{c} D^{T}=\frac{F^{T-i}}{F^{T}-F^{T-i}}. \end{array}$$

Sometimes, adding or removing hidden nodes will not do the trick, so consider adding or removing a hidden layer. According to the empirical formula, the position and node number of the new hidden layer generally increase between the final hidden layer and the output layer, and its dimension is set as

(3) $$\begin{array}{c} N_{\text{new}}=\frac{\mathrm{int}\left[\log_{2}\left(N_{K}+N_{K-1}\right)\right]}{N}. \end{array}$$

Given a nonlinear mapping from *R*_3_ to *R*_2_,

(4) $$\begin{array}{c} f=\left\{\begin{array}{c} y_{1}=\frac{e^{x2}-e^{x1}}{2},\\ y_{2}=\frac{x_{3}^{2}-x_{2}^{2}}{2}. \end{array}\right) \end{array}$$

The learning algorithm uses the sample calculation error index as the convergence judgment condition and takes the convergence threshold of the network structure learning error as *E*_0_ = 0.0008. Population evolution period (*T*) is the period of population level evolution operation relative to individual level evolution operation within the population, which is generally expressed by the positive integer of individual level evolution algebra [14].

(5) $$\begin{array}{c} D\left(t\right)=\frac{f_{\max}\left(t\right)}{f_{\max}\left(t+T\right)-f_{\max}\left(t-T\right)}, \end{array}$$

where *f*_max_ (*t*) represents the adaptive value of the optimal individual of the population at time *T*.

### 3.3. Landscape Planning Technical Route

Plants, as one of the basic components of the ecosystem, are also one of the important factors of landscape vision and are the most active and critical factors in the creation of habitats such as parks. It directly affects the quality of the landscape. Wetland plants are a transitional type between land plants and aquatic plants and have the characteristics of adapting to semiwater and semiland environment. For plant landscape planning and design, the landscape area should retain the existing vegetation as much as possible according to the existing vegetation types and overall layout requirements. This not only ensures the diversity of habitats but also pursues the creation of a different forest plant landscape change so that the diversity of the park's wetland ecosystem and the diversity of the landscape can be fully displayed.

In the development of plant landscape planning and design of landscape architecture, in order to fully achieve the actual effect of plant landscape design, we need to pay attention to several aspects. First of all, before the implementation of the relevant planning and design work, it is necessary to fully understand the requirements of the relevant plant landscape, collect the planning and design information of the plant landscape with reference significance more comprehensively, and ensure the smoothness of the later work. Secondly, it is necessary to conduct field research in the planning area of the scenic forest park, fully understand the climate and geomorphology of the relevant area, soil conditions, and other conditions, conduct a comprehensive analysis of this information, select suitable landscape plants in the area, and lay a foundation for the subsequent plant landscape design. Finally, it is necessary to carry out a detailed investigation of the surrounding areas of the landscaped garden, to provide a reference for the subsequent plant landscape design, and then effectively ensure the coordination of the plant landscape and surrounding plants in the landscaped garden.

This study focuses on theoretical research and appropriately combines case analysis. On the basis of scientific and comprehensive data collection, classification and induction, field investigation, theoretical analysis, case study, and other forms of in-depth understanding of the research object, use landscape, planning, architecture, geography, sociology, ecology, art, and other pieces of multidisciplinary knowledge. The technical route of this landscape planning is shown in Figure 2.

In the actual plant landscape planning and design of landscape architecture, in addition to the overall concept design, relevant personnel also need to draw a detailed construction drawing, according to the requirement of the relevant party at the same time, a detailed comparison of various construction aspects, and choose a satisfying effect design and conform to the economic benefit and practical construction design. In the process of drawing the specific construction design drawings, the plant species and transplant sites of each construction area should be marked in detail. At the same time, the plant names, attention points, and specific transplant construction measures should be clearly indicated, so as to effectively ensure the survival rate of plant transplantation. In the specific construction drawings, the location data such as the transplant spacing of different plants and the position relationship between them and other landscapes should be marked according to the effect design, and the traceable identification method should be adopted to improve the efficiency of the plant transplant construction process. It can take multiview detailed drawing design, such as plan, elevation, and node diagram, to provide detailed and reliable construction drawings for the construction personnel.

## 4. Results and Analysis

### 4.1. Landscape Green Space Layout and Plant Species Analysis

The planned greening area of the virtual landscape covers 5060 hectares, including 4621.44 hectares of built-up area. There are 12 parks, the park area of 693.91 hectares and annual visitor of 3.32 million person-times. The city's per capita public green area is 9.55 square meters, the green rate of the built-up area is 25.39%, and the green coverage rate of the built-up area is 33.42%. In the green space structure, public green space is 994 hm^2^, unit affiliated green space is 428.36 hm^2^, residential green space is 83.98 hm^2^, production green space is 765 hm^2^, protection green space is 1237 hm^2^, road green space is 143 hm^2^, and scenic forest land is 972 hm^2^ (Figures 3 and 4).

From the process of ecological garden construction, we can see that we need to pay more attention to the principle of plant diversity. The number and number of actual species and the corresponding biological relationship can effectively highlight the characteristics of ecological balance. In different natural environments, abundant and stable plant abundance can ensure the stability of the ecological environment and make the natural environment have more opportunities for sustainable development. From the perspective of biological theory, it can make ecological gardens achieve sustainable development and maintain diversity, which is also an important prerequisite for maintaining the appreciation of ecological gardens and can show an irreplaceable role.

A total of 114 species of plants were recorded in the study area. In the field investigation, they mainly included algae, fungi, lichens, bryophytes, ferns, gymnosperms, and angiosperms, which were divided into trees, shrubs, vines, and herbs according to the morphology of stems. The classification and quantity distribution are shown in Figure 5.

As can be seen from Figure 5, the growth process and growth changes of different plants have different seasonal characteristics, but these characteristics are relatively fixed in a fixed area. Botanically speaking, the landscape of plants can be said to change from day to day as plants grow. The changes are subtle over a short period of time and are difficult to detect directly. However, in the seasonal changes of plant growth, such changes are relatively prominent, which is also an important reason for the ornamental nature of plants. This seasonal change is not only the form and color but also an important embodiment of seasonal climate change. In planning and design, plant landscape designers should make scientific and reasonable allocation according to the timing of different plants in the seasonal changes to form a unique planning and design scheme. The so-called timing is based on the natural growth cycle of plants in nature (one year as a unit). The growth, flowering, and fruit bearing of plants are completed in different seasons and different time periods, which is also an important characteristic basis of plant diversity. In this natural law, designers should carry out reasonable planning and design according to the flowering time sequence of different plants, in order to achieve the most ornamental and aging plant landscape, so as to add beautiful color landscape to the overall aesthetic effect of the landscaped garden.

### 4.2. Multispecies Plant Landscape Planning Model

The distribution and prediction of multispecies plants are the main decision-making basis of landscape planning. Traditional models such as the time series method and regression analysis method are difficult to modify and do not have self-learning ability, so it is difficult to meet the requirements of accuracy. The neural network model can better solve the problems faced by traditional methods [6]. The key to improve the global convergence rate of the multimodal function optimization problem is to guide the population to search the global optimal peak quickly. In this algorithm, a series of local peaks given in the process of mature population evolution can guide the algorithm to search more effectively. For MLP or RBF model, it can be known from prior knowledge that if the optimal individual of a certain group cannot meet the accuracy requirements of the model after maturity and convergence, it can be regarded as the “lowest structural complexity” of the model solution, and conversely, it can be regarded as the “highest structural complexity” model. This method can be used to guide the direction of out-of-species evolution and avoid the search area of invalid population gene. Compared with the general evolutionary design method, this method can effectively improve the global convergence rate. Using the multispecies evolutionary genetic algorithm proposed in this paper, a neural network model with good structure and weight is constructed automatically by training and verifying the historical data samples. By analyzing the error between real data and forecast data, the model can be revised effectively. The data of the multispecies evolutionary training process of neural networks are shown in Figures 6 and 7. The variation of species richness along environmental gradient is still an important factor affecting landscape design, and understanding the general determinants of species richness is particularly important for species conservation. There are two main factors affecting species richness: environmental factors and biological factors. The influence of environmental factors on species richness is not necessarily direct but may also be indirect through influencing other biological factors.

### 4.3. Negative Sampling Effect Test Results

When planning and designing the plant landscape of landscape architecture, we should use the strategy of conceptual planning, analyze the status quo of prebuilt landscape architecture through conceptual planning, set the planning and design goals of landscape architecture, combine these goals to do a good job in the multidimensional planning and design of landscape architecture, and design more details of landscape architecture accordingly. Landscape architects should be clear about the requirements and regulations of planning and objectives and do a detailed and multidimensional conceptual design of plant landscape according to the planning. Overall, it covers feature planning, time planning, and space planning. First, regarding feature planning, in the process of conceptual planning of plant landscape, characteristic planning is a key content. Designers should combine the overall planning of landscape architecture to design featured landscapes, highlighting the overall characteristics of various plant landscapes and landscape architecture on the whole, and then make it present a more ideal design effect. Second, regarding time planning, optimized time planning is of great significance in the design of plant landscapes. Combining the specific status and corresponding changes of various plants in each season, this paper designs targeted planning to adapt to different seasons, thereby presenting plant landscapes of different colors and enhancing the practicality and ornamentalness of plant landscapes. Thirdly, Regarding space planning, from the perspective of space planning, plant landscape construction space usually occupies a larger area in landscaped gardens. Therefore, it is necessary to reasonably plan the specific space layout of plant landscape and the collocation of different types of plant landscape to effectively improve the design quality of landscape architecture.

The random distribution of plant populations from the 2020 survey was tested. As can be seen from Figure 7, more than one-third of the observed values of shrubs are not covered by species richness (including standard deviation), indicating that “negative sampling” has no impact on plant species richness. Similarly, Figure 8 shows that the species richness of plants is not affected by “negative sampling.”

In this study, eight test points were selected and the distribution of plant species was investigated, as shown in Figure 9. Based on the above rules, we use Monte Carlo sampling to generate 500 sets of models, each with a unique combination of parameter values. By this sampling method, the parameters have representative values in their respective ranges. After obtaining the running results of 500 sets of models, we calculated the coefficient of determination between each parameter and the species concentration of each model and quantified the explanatory variance of each parameter to the model output results. All parameters are then sorted and the most sensitive parameters are selected for subsequent optimization.

The parameters of the genetic algorithm include population size, crossover probability, mutation probability, and maximum number of iterations (Figure 10). In this study, these four parameters were set to 20, 0.60, 0.10, and 1000, respectively. In this optimization algorithm, individual representatives in the genetic algorithm were set up with CoSiNE models with different ecological parameter values. The parameter values were compiled in real code, the cost function *F* was used to refer to the fitness in the algorithm, and the *F* value represented the difference between the model results and the observed values. The genetic individuals of each generation were selected using the roulette model. A combination of parameters with better performance is generated according to the set crossover and mutation probabilities. The whole optimization process is to further reduce the cost function until the desired effect is met. The expected optimal setting is related to the optimal fitness value or the maximum number of iterations.

## 5. Conclusion

A good plant landscape is conducive to beautifying the ecological environment of a landscaped garden, displaying the garden style, improving the living atmosphere, and providing leisure and entertainment. Aiming at the lack of general neural network modeling and effective design methods, this paper puts forward the evolution genetic algorithm, gives the evolutionary neural network structure design method based on this method, compared with the general ANN structure learning algorithm method, and can use the shorter encoded representation of the neural network structure and weights and relatively simple structure and training rules. The contradiction between search space and evolution rules is solved, and the structure and weight can be optimized. This model combines the specific states and corresponding changes of various plants in each season to design targeted planning, which can adapt to different seasons, present different colors of plant landscape, and then promote the practicality and appreciation of plant landscape. Thirdly, from the perspective of space planning, plant landscape construction space usually occupies a larger area in the landscaped garden. Therefore, it is necessary to reasonably plan the specific space layout of plant landscape and the collocation of different types of plant landscape to effectively improve the design quality of landscape architecture. Through the analysis of the application of the genetic algorithm in landscape design practice, it can be found that this technology not only effectively improves the quality and efficiency of design work but also plays an important role in broadening the design idea and optimizing the design concept. Combined with the specific development, it can be predicted that, in the following landscape design process, the application and promotion of the genetic algorithm model will move to a new height. It is necessary to adhere to the correct concept of plant landscape design, optimize the design strategy, and design diversified plant landscapes that are compatible with the local customs, geographical environment, climate, and geology. It is also necessary to fully integrate the excellent cultural elements of traditional construction and design of landscape architecture. Through the proper collocation and reasonable selection of different plants, the cultural taste, practical effect, and aesthetic degree of landscape architecture can be effectively strengthened.

## Figures and Tables

**Figure 1:** Elements and layout of landscape planning.

**Figure 2:** Framework design of diversified plant landscape planning based on neural network algorithm.

**Figure 3:** The distribution of green space in the planned area.

**Figure 4:** Plant distribution in the five areas of the planning area.

**Figure 5:** Species and number of plant species in the area.

**Figure 6:** Optimal network structure for multispecies evolutionary training of neural networks.

**Figure 7:** Optimal check error, optimal training error, and learning efficiency of multispecies evolutionary training of neural networks.

**Figure 8:** The predicted value and scatter distribution of plant species richness in the planned areas.

**Figure 9:** The number of specific species of plants in each of the 8 zones marked.

**Figure 10:** Comparison of test results of the neural network model in multispecies plant landscape planning and design projects.

## Data Availability

The data used to support the findings of this study are available from the corresponding author upon request.
